The article "Fuzzy Stress-Strength Model and Mean Remaining Strength for Lindley Distribution: Estimation and Application in Cancer of Benign Endocrine" was published in 2023. Journal: Comput Math Methods Med.

# Fuzzy Stress-Strength Model and Mean Remaining Strength for Lindley Distribution: Estimation and Application in Cancer of Benign Endocrine

**DOI:** 10.1155/2023/8952946

**Published:** 2023-11-02

**Authors:** Marwa K. H. Hassan, Abdisalam Hassan Muse

**Affiliations:** ^1^Department of Mathematics, Faculty of Education, Ain Shams University, Cairo, Egypt; ^2^Faculty of Science and Humanities, School of Postgraduate Studies and Research (SPGSR), Amoud University, Borama 25263, Somalia

## Abstract

This paper is interested in the Bayesian and non-Bayesian estimation of the stress-strength model and the mean remaining strength when there is fuzziness for stress and strength random variables having Lindley's distribution with different parameters. A fuzzy is defined as a function of the difference between stress and strength variables. In the context of Bayesian estimation, two approximate algorithms are used importance sampling algorithm and the Monte Carlo Markov chain algorithm. For non-Bayesian estimation, maximum likelihood estimation and maximum product of spacing method are used. The Monte Carlo simulation study is performed to compare between different estimators for our proposed models using statistical criteria. Finally, to show the ability of our proposed models in real life, real medical application is introduced.

## 1. Introduction

Lindley [1, 2] introduced the Lindley distribution in the context of Bayesian statistics, Ghitany et al. [3] studied the statistical properties of the Lindley distribution, and they showed that it is better than the exponential distribution because it has an increasing hazard rate function. This is the main reason to perform this study about the Lindley distribution. Shanker et al. [4] made a comparative study between the Lindley distribution and exponential distribution for various lifetime data in many fields such as biomedical science and engineering, and they found that the Lindley distribution is better than the exponential distribution.

**Definition 1 .**

A random variable *X* is said to have the Lindley distribution with parameter *θ*. If its probability density function is given by

(1) $$\begin{array}{c} f\left(x;\theta \right)=\frac{\theta^{2}}{\theta +1}\;\left(1+x\right)e^{-\theta \;x}\;x>0,\theta >0. \end{array}$$

The cumulative distribution function is given by

(2) $$\begin{array}{c} F\left(x;\theta \right)=1-\left(1+\frac{\theta }{1+\theta }\;x\right)e^{-\theta \;x}. \end{array}$$

The hazard rate function is given by

(3) $$\begin{array}{c} h\left(x;\theta \right)=\frac{\theta^{2}\;\left(1+x\right)}{1+\theta \;\left(1+x\right)}, \end{array}$$

and the mean residual function is given by

(4) $$\begin{array}{c} \mu \left(x\right)=E\left[X-x\left|X>x\right.\right]=\frac{1}{\theta }+\frac{1}{\theta \left(1+\theta +\theta \;x\right)}. \end{array}$$

Ghitany et al. [3] proved that the Lindley distribution is unimodal for 0 < *θ* < 1 as shown in Figure 1, decreasing for *θ* ≥ 1 as shown in Figure 2, and *μ*(*x*) is decreasing for *X* as shown in Figure 3.

The article "Fuzzy Stress-Strength Model and Mean Remaining Strength for Lindley Distribution: Estimation and Application in Cancer of Benign Endocrine" was published in 2023. Journal: Comput Math Methods Med.

Since most of the engineering processes inherently have uncertainty that must be dealt with and represented effectively, sometimes, the data cannot be reported precisely under some unexpected situations that can occur by misdetection of failures by a user, by inattentive records or measurements, etc. In addition, the subjective evaluation of the lifetime data leads to the fuzziness. So, the main aim of this paper is to study the fuzzy stress-strength model and fuzzy mean remaining strength when the stress and strength variables are independent having Lindley's distribution with different shape parameters *θ*. Now, we introduce an overview about stress-strength model, mean remaining strength, and fuzzy function. The fuzzy function is defined as a function of the difference between stress-strength variables, and it makes more sensitive analysis, see [5] and Eryilmaz and Tutuncu [6]. So, it encourages us to make this study to compare the behavior of the stress-strength model and mean remaining strength in both cases, the existence and nonexistence of fuzziness. The stress-strength models have an important role in many fields such as engineering, quality control, medicine, and economic. The reliability parameter is *R* = *P*[*Y* < *X*], where *X* is the strength random variable and *Y* is the stress random variable. In the reliability analysis, *R* describes the life of a component that has strength variable *X* and is subjected to random variable stress *Y*. The system fails if and only if the stress is greater than the strength. The stress-strength models have been studied by many authors; for references in the past, see Kotz et al. [7]. For the Lindley distribution, see Al-Mutairi et al. [8] and Hassan [9]. Also, there are many references for other distributions such as the beta Gompertz distribution, see Hassan [10], and the exponential Pareto distribution, see Al-Omari et al. [11]. In the context of the mean remaining strength (MRS) of the component as the expected remaining strength under the stress, see Gurler [12], Gurler et al. [13], Bairamove et al. [14], and Kizilaslan [15]. Fuzziness is introduced in reliability by Huang [5]. In recent, Eryilmaz and Tutuncu [6] introduced the stress-strength reliability in the presence of fuzziness, Sabry et al. [16] introduced fuzzy reliability for inverse Rayleigh distribution, and Yazgan et al. [17] introduced the fuzzy stress-strength model for weight exponential distribution and also introduced the fuzzy mean remaining strength for the same distribution. This paper is organized as follows: there is a fuzzy stress-strength model and a fuzzy mean remaining strength when the stress and strength are two independent Lindley distributions with different shape parameters in Section 2; in Section 3, non-Bayesian estimation of fuzzy stress-strength model and fuzzy mean remaining strength using maximum likelihood estimation (MLE) method and the maximum product of the spacing estimation (MPS) method; in Section 4, Bayesian estimation using importance sampling algorithm (IS) and Monte Carlo Markov chain algorithm (MCMC). The Monte Carlo simulation study is constructed to compare between different estimators for our proposed models in Section 5. Real application is introduced to show the validity of our proposed model in real life in Section 6. Finally, in Section 7, we conclude the results of our paper.

The article "Fuzzy Stress-Strength Model and Mean Remaining Strength for Lindley Distribution: Estimation and Application in Cancer of Benign Endocrine" was published in 2023. Journal: Comput Math Methods Med.

## 2. Fuzzy Stress-Strength Model (FSS) and Fuzzy Mean Remaining Strength (FMRS)

In this section, we introduce the FSS model and FMRS when the stress and strength variables are independent and have Lindley's distribution with different shape parameters.

### 2.1. FSS Model for Lindley Distribution

Al-Mutairi et al. [8] introduced a classical stress-strength model when the stress (*Y*)and strength (*Y*)variables are independent and have Lindley's distribution with different shape parameters *θ*_2_ and *θ*_1_, respectively, as follows:

(5) $$\begin{array}{c} R=P\left[Y<X\right]=\iint_{y<x}^{\infty }dF_{X}\left(x\right)dF_{Y}\left(y\right)=\frac{\theta_{2}^{2}\left(2\theta_{1}+\left(1+2\theta_{1}\right)\left(\theta_{1}+\theta_{2}\right)+\left(1+\theta_{1}\right){\left(\theta_{1}+\theta_{2}\right)}^{2}\right)}{\left(1+\theta_{1}\right)\left(1+\theta_{2}\right){\left(\theta_{1}+\theta_{2}\right)}^{3}}. \end{array}$$

Eryilmaz and Yutuncu [6] defined the FSS model as

(6) $$\begin{array}{c} \text{FSS}=P\left[Y<X\right]=\iint_{y<x}^{\infty }\mu_{A\left(y\right)}\left(x\right)\;dF_{X}\left(x\right)dF_{Y}\left(y\right), \end{array}$$

where

(7) $$\begin{array}{c} \mu_{A\left(y\right)}\left(x\right)=\left\{\begin{array}{cc} 0 & \&y\geq x\\ 1-e^{-k\left(x-y\right)} & y<x \end{array}.\right. \end{array}$$

Hence, in the case of the Lindley distribution, we defined FSS as

(8) $$\begin{array}{c} \text{FSS}=\iint_{y<x}^{\infty }\left(1-e^{-k\left(x-y\right)}\right)\left(\frac{\theta_{1}^{2}}{1+\theta_{1}}\;\left(1+x\right)e^{-\theta_{1}x}\right)\left(\frac{\theta_{2}^{2}}{1+\theta_{2}}\;\left(1+y\right)e^{-\theta_{2}y}\right)\text{dxdy}, \end{array}$$

(9) $$\begin{array}{c} \text{FSS}=\frac{k\theta_{2}^{2}\left(\theta_{1}\left(3k+\theta_{1}\left(4+3k+\theta_{1}\left(4+k+\theta_{1}\right)\right)\right)+\left(k+2\theta_{1}\left(1+2k+\theta_{1}\left(3+k+\theta_{1}\right)\right)\right)\theta_{2}+\left(k+\theta_{1}\left(2+k+\theta_{1}\right)\right)\theta_{2}^{2}\right)}{\left(1+\theta_{1}\right){\left(k+\theta_{1}\right)}^{2}\left(1+\theta_{2}\right){\left(\theta_{1}+\theta_{2}\right)}^{3}}. \end{array}$$

We note that the classical stress-strength model is greater than the fuzzy stress-strength model, but for large *k*, the fuzzy model approximately equals the classical model.

The article "Fuzzy Stress-Strength Model and Mean Remaining Strength for Lindley Distribution: Estimation and Application in Cancer of Benign Endocrine" was published in 2023. Journal: Comput Math Methods Med.

Figure 4 shows the classical stress-strength model for different values of *θ*_1_ and *θ*_2_. Also, Figure 5 shows fuzzy stress-strength model for different values of *k*, *θ*_1_ and *θ*_2_.

### 2.2. FMRS for Lindley Distribution

Gurler [12] defined the mean remaining strength (MRS)as

(10) $$\begin{array}{c} \text{MRS}=E\left[X-Y\left|Y<X\right.\right]=\int_{0}^{\infty }\left(\frac{\int_{0}^{\infty }\int_{x+y}^{\infty }dF_{X}\left(x\right)dF_{y}\left(y\right)}{P\left[Y<X\right]}\right)\text{dx}. \end{array}$$

Then, we use this definition to get MRS for the Lindley distribution as

(11) $$\begin{array}{c} \text{MRS}=\frac{\theta_{1}{\left(2+\theta_{1}\right)}^{2}+2\left(1+\theta_{1}\left(3+\theta_{1}\right)\right)\theta_{2}+\left(2+\theta_{1}\right)\theta_{2}^{2}}{\theta_{1}\left(2\theta_{1}+\left(1+2\theta_{1}\right)\left(\theta_{1}+\theta_{2}\right)+\left(1+\theta_{1}\right){\left(\theta_{1}+\theta_{2}\right)}^{2}\right)}. \end{array}$$

Yazgan et al. [17] defined fuzzy mean remaining strength as

(12) $$\begin{array}{c} \text{FMSR}=\int_{0}^{\infty }\left(\frac{\int_{0}^{\infty }\int_{x+y}^{\infty }\mu_{A\left(y\right)}\left(x\right)dF_{X}\left(x\right)dF_{y}\left(y\right)}{FSS}\right)\text{dx}. \end{array}$$

Then, we can get FMRS for the Lindley distribution as

(13) $$\begin{array}{c} \text{FMSR}=\frac{\theta_{1}\left(4k^{2}+\theta_{1}\left(4k\left(3+k\right)+\theta_{1}\left(10+k\left(12+k\right)+\theta_{1}\left(10+3k+2\theta_{1}\right)\right)\right)\right)+2\left(k^{2}+\theta_{1}\left(3k\left(1+k\right)+\theta_{1}\left(3+k\left(9+k\right)+\theta_{1}\left(8+3k+2\theta_{1}\right)\right)\right)\right)\theta_{2}+\left(2k^{2}+\theta_{1}\left(k+\theta_{1}\right)\left(6+k+2\theta_{1}\right)\right)\theta_{2}^{2}}{\theta_{1}\left(k+\theta_{1}\right)\left(\theta_{1}\left(3k+\theta_{1}\left(4+3k+\theta_{1}\left(4+k+\theta_{1}\right)\right)\right)+\left(k+2\theta_{1}\left(1+2k+\theta_{1}\left(3+k+\theta_{1}\right)\right)\right)\theta_{2}+\left(k+\theta_{1}\left(2+k+\theta_{1}\right)\right)\theta_{2}^{2}\right)}. \end{array}$$

The article "Fuzzy Stress-Strength Model and Mean Remaining Strength for Lindley Distribution: Estimation and Application in Cancer of Benign Endocrine" was published in 2023. Journal: Comput Math Methods Med.

## 3. Non-Bayesian Estimation of FSS and FMRS

In this section, we discuss the maximum likelihood estimation method (MLE) and the maximum product of the spacing estimation (MPS) for *R*, MRS, FSS, and FMRS.

### 3.1. MLE of FSS and FMRS

Let *X*_1_ ⋯ *X*_*n*_ be a random sample of size *n* from the Lindley distribution with shape parameter *θ*_1_ and *Y*_1_ ⋯ *Y*_*n*_ be a random sample of size *m* from the Lindley distribution with parameter *θ*_2_. Then, the maximum likelihood estimators of *θ*_1_ and *θ*_2_ are given by

(14) $$\begin{array}{c} {\hat{\theta }}_{1}=\frac{-\left(\bar{x}-1\right)+\sqrt{{\left(\bar{x}-1\right)}^{2}+8\bar{x}}}{2\;\bar{x}},\;\bar{x}=\frac{1}{n}\overset{n}{\underset{i=1}{\sum }}x_{i},\\ {\hat{\theta }}_{2}=\frac{-\left(\bar{y}-1\right)+\sqrt{{\left(\bar{y}-1\right)}^{2}+8\bar{y}}}{2\;\bar{y}},\;\bar{y}=\frac{1}{m}\overset{m}{\underset{j=1}{\sum }}y_{j}. \end{array}$$

For more details, see Ghitany et al. [3]. Use the invariance property of MLE to get the estimators of *R*, MRS, FSS, and FMRS by replacing *θ*_1_ and *θ*_2_ by its maximum likelihood estimators ${\hat{\theta }}_{1}$and${\hat{\theta }}_{2}$in equations (5), ((8)), ((11)), and ((13)) and denoted by$\hat{R},\hat{\text{MRS}},\hat{\text{ FSS}},$and$\hat{\text{FMRS}}$.

### 3.2. MPS Estimation of FSS and FFMRS

First, we introduce an overview for MPS estimation as follows: let *X*_1_ ⋯ *X*_*n*_ be a random sample of size *n* from a population with distribution parameter *θ*. Then, the spacing is defined as the gap between two distinct distribution functions as follows:

(15) $$\begin{array}{c} D_{i}\left(\theta \right)=F\left(x_{i};\theta \right)-F\left(x_{i-1};\theta \right)\;i=1\cdots n+1, \end{array}$$

where ∑_*i*=1_^*n*^*D*_*i*_(*θ*) = 1 and *D*_*i*_(*θ*) are defined as for *x*_1:*n*_ ⋯ *x*_*n*:*n*_.

(16) $$\begin{array}{c} D_{i}\left(\theta \right)=\left\{\begin{array}{c} D_{1}\left(\theta \right)=F\left(x_{1:n};\theta \right)\\ D_{i}\left(\theta \right)=F\left(x_{i:n};\theta \right)-F\left(x_{i-1:n};\theta \right)\\ D_{n+1}\left(\theta \right)=1-F\left(x_{n:n};\theta \right) \end{array}.\right. \end{array}$$

The maximum spacing estimator of the parameter *θ* is defined as the value that maximizes the logarithm of the geometric mean of a sampling spacing, see [18].

(17) $$\begin{array}{c} \hat{\theta }=\arg\max S_{n}\left(\theta \right), \end{array}$$

where *S*_*n*_(*θ*) = *Ln*[∏_*i*=1_^*n*^*D*_*i*_(*θ*)]^1/*n*+1^.

Now, we use the MPS estimation method to get the estimators of *R*, MRS, FSS, and FMRS as follows: let *X*_1_ ⋯ *X*_*n*_ be a random sample of size *n* from the Lindley distribution with shape parameter *θ*_1_ and *Y*_1_ ⋯ *Y*_*n*_ be a random sample of size *m* from the Lindley distribution with parameter *θ*_2_. Then,

(18) $$\begin{array}{c} S_{n,m}\left(\theta_{1},\theta_{2}\right)=Ln{\left[\overset{n}{\underset{i=1}{\prod }}D_{i}\left(\theta_{1}\right)\right]}^{1/n+1}\;{\left[\overset{m}{\underset{j=1}{\prod }}D_{j}\left(\theta_{2}\right)\right]}^{1/m+1}=\frac{1}{n+1}\left[Ln\left(D_{1}\left(\theta_{1}\right)\right)+Ln\left(D_{n+1}\left(\theta_{1}\right)\right)+\overset{n}{\underset{i=2}{\sum }}Ln\left(D_{i}\left(\theta_{1}\right)\right)\right]+\frac{1}{m+1}\left[Ln\left(D_{1}\left(\theta_{2}\right)\right)+Ln\left(D_{m+1}\left(\theta_{2}\right)\right)+\overset{m}{\underset{j=2}{\sum }}Ln\left(D_{j}\left(\theta_{2}\right)\right)\right]. \end{array}$$

To get the maximum spacing estimators for *θ*_1_ and *θ*_2_ denoted by *θ*_1_^MPS^ and *θ*_2_^MPS^, respectively, maximize *S*_*n*,*m*_(*θ*_1_, *θ*_2_) using an optimization algorithm and using the invariance property of MLE to get the estimators of*R*, MRS, FSS, and FMRS by replacing *θ*_1_ and *θ*_2_ by its maximum likelihood estimators *θ*_1_^MPS^ and *θ*_2_^MPS^ in equations (8), ((11)), ((13)), and ((18)) which are denoted by *R*^MPS^, MRS^MPS^, FSS^MPS^, and FMRS^MPS^.

The article "Fuzzy Stress-Strength Model and Mean Remaining Strength for Lindley Distribution: Estimation and Application in Cancer of Benign Endocrine" was published in 2023. Journal: Comput Math Methods Med.

## 4. Bayesian Estimation of FSS and FMRS

In this section, we obtain the Bayesian estimators of *R*, MRS, FSS, and FMRS based on the Lindley distribution. Let *θ*_1_ and *θ*_2_ be two independent random variables with gamma prior distribution where *θ*_1_ ≈ Gamma(*a*_1_, *b*_1_) and *θ*_2_ ≈ Gamma(*a*_2_, *b*_2_) [19–21]. Then, the joint prior distribution of *θ*_1_ and *θ*_2_ is

(19) $$\begin{array}{c} L\left(X,Y\left|\theta_{1},\theta_{2}\right.\right)\propto \frac{\theta_{1}^{2n}\;\theta_{2}^{2\;m}}{{\left(1+\theta_{1}\right)}^{n}\;{\left(1+\theta_{2}\right)}^{m}}\;e^{\left(-\theta_{1}\;\overset{n}{\underset{i=1}{\sum }}x_{i}-\theta_{2}\overset{m}{\underset{j=1}{\sum }}y_{j}\right)}. \end{array}$$

And the posterior density function of *θ*_1_ and *θ*_2_ is given by

(20) $$\begin{array}{c} L\left(\theta_{1},\theta_{2}\left|X,Y\right.\right)=\frac{c}{{\left(1+\theta_{1}\right)}^{n}\;{\left(1+\theta_{2}\right)}^{m}}\;\Gamma \left(\theta_{1};a_{1}+2\;n-1,b_{1}+\overset{n}{\underset{i=1}{\sum }}x_{i}\right),\\ \Gamma \left(\theta_{2};a_{2}+2\;m-1,b_{2}+\overset{m}{\underset{j=1}{\sum }}y_{j}\right), \end{array}$$

where *C* is the normalizing constant. Now, the Bayes estimator for any function Ψ  of *θ*_1_ and *θ*_2_ is given by

(21) $$\begin{array}{c} \Psi_{\text{Bayes}}\left(\theta_{1},\theta_{2}\right)=\frac{\int_{0}^{\infty }\int_{0}^{\infty }\Psi \left(\theta_{1},\theta_{2}\right)L\left(\theta_{1},\theta_{2}\left|X,Y\right.\right)d\theta_{1}d\theta_{2}}{\int_{0}^{\infty }\int_{0}^{\infty }L\left(\theta_{1},\theta_{2}\left|X,Y\right.\right)d\theta_{1}d\theta_{2}}. \end{array}$$

But we cannot compute the analytic form of  Ψ_Bayes_. Then, we must consider some approximations such as the Lindley approximation, importance sampling (IS) techniques, and the Monte Carlo Markov chain (MCMC) algorithm. In this study, we are interested in IS algorithm and MCMC algorithm.

The article "Fuzzy Stress-Strength Model and Mean Remaining Strength for Lindley Distribution: Estimation and Application in Cancer of Benign Endocrine" was published in 2023. Journal: Comput Math Methods Med.

### 4.1. IS Algorithm

IS algorithm is introduced by Kloek and Dijk [22]. To use this algorithm, get the Bayesian estimators of *R*, MRS, FSS, and FMRS as follows:

1. Suppose that *θ*_1_ ≈ Gamma(*a*_1_, *b*_1_) and *θ*_2_ ≈ Gamma(*a*_2_, *b*_2_) be independent random variables
2. Generate *θ*_11_ ≈ Γ(*θ*_1_; *a*_1_ + 2 *n* − 1, *b*_1_ + ∑_*i*=1_^*n*^*x*_*i*_) and *θ*_21_ ≈ Γ(*θ*_2_; *a*_2_ + 2 *m* − 1, *b*_2_ + ∑_*j*=1_^*m*^*y*_*j*_)
3. Repeat step 2 *N*-times to obtain (*θ*_11_, *θ*_21_) ⋯ (*θ*_1*N*_, *θ*_2*N*_)
4. The Bayesian estimator of any function Ψ(*θ*_1_, *θ*_2_) is given by

(22) $$\begin{array}{c} \Psi_{\text{Bayes}}^{\text{IS}}\left(\theta_{1},\theta_{2}\right)=\overset{N}{\underset{i=1}{\sum }}W_{i}\;\Psi_{i}\left(\theta_{1},\theta_{2}\right), \end{array}$$

where *W*_*i*_ = *h*(*θ*_1*i*_, *θ*_2*i*_)/∑_*i*=1_^*N*^*h*(*θ*_1*i*_, *θ*_2*i*_) and *h*(*θ*_1*i*_, *θ*_2*i*_) = 1/(1 + *θ*_1*i*_)^*n*^ (1 + *θ*_2*i*_)^*m*^.

### 4.2. MCMC Algorithm

In this subsection, we use the MCMC algorithm to get the Bayesian estimators of *R*, MRS, FSS, and FMRS based on the Lindley distribution; the MCMC algorithm using the Gibbs simpler; and the Metropolis-Hastings algorithm (MH); for more details about MH algorithm, see [23]. Now, to get the Bayesian estimators of *R*, MRE, FSS, and FMRS using the following algorithm,

1. Let the noninformative prior of *θ*_1_ and *θ*_2_ as ∏_*i*_(*θ*_*i*_) ∝ *θ*_*i*_^−1^ *i* = 1, 2. For more details about the noninformative, see [24, 25]
2. The joint posterior distribution *θ*_1_ and *θ*_2_ is

(23) $$\begin{array}{c} L\left(\theta_{1},\theta_{2}\left|X,Y\right.\right)=k\;\frac{\theta_{1}^{2n-1}\;\theta_{2}^{2\;m-1}}{{\left(1+\theta_{1}\right)}^{n}\;{\left(1+\theta_{2}\right)}^{m}}\;e^{\left(-\theta_{1}\;\overset{n}{\underset{i=1}{\sum }}x_{i}-\theta_{2}\overset{m}{\underset{j=1}{\sum }}y_{j}\right)}\;\overset{n}{\underset{i=1}{\prod }}\left(1+x_{i}\right)\overset{m}{\underset{j=1}{\prod }}\left(1+y_{j}\right) \end{array}$$

(3) Let the start values *θ*_1_^(0)^ and *θ*_2_^(0)^ for *θ*_1_ and *θ*_2_, respectively
(4) Generate *θ*_1_^(*k*)^ from *π*(*θ*_1_|*X*) ∝ (*θ*_1_^(2 *n* − 1)^/(1 + *θ*_1_)^*n*^) *e*^−*θ*_1_∑_*i*=1_^*n*^*x*_*i*_^ ∏_*i*=1_^*n*^(1 + *x*_*i*_)
(5) Generate *θ*_2_^(*k*)^ from *π*(*θ*_2_|*Y*) ∝ (*θ*_2_^(2 *m* − 1)^/(1 + *θ*_2_)^*m*^) *e*^−*θ*_2_∑_*j*=1_^*m*^*y*_*j*_^ ∏_*j*=1_^*m*^(1 + *y*_*j*_)
(6) Repeat steps 4 and 5 *M*-times
(7) Compute the Bayes estimator for any function Ψ(*θ*_1_, *θ*_2_) which is given by

(24) $$\begin{array}{c} \Psi_{\text{Bayes}}^{\text{MCMC}}\left(\theta_{1},\theta_{2}\right)=\frac{1}{M-M_{0}}\;\overset{M}{\underset{k=M_{0}+1}{\sum }}\Psi \left(\theta_{1}^{\left(k\right)},\theta_{2}^{\left(k\right)}\right) \end{array}$$

where *M*_0_ is the burn-in period of the generated Markov chain.

The article "Fuzzy Stress-Strength Model and Mean Remaining Strength for Lindley Distribution: Estimation and Application in Cancer of Benign Endocrine" was published in 2023. Journal: Comput Math Methods Med.

## 5. Monte Carlo Simulation Study

In this section, we construct a Monte Carlo simulation study to investigate the behavior of different estimates for *R*, MRS, FSS, and FMRS. All calculations for this study are performed using R-program using different packages (*nlme*, *likelihood*, *LindleyR*, *MASS*, *STAT4*, *EstimatomTools*, *BMT*, *MCMC*, and *fitdistplus)*. Also, we compare the different estimates of *R*, MRS, FSS, and FMRS for different values of *k*, sample size, and different values of distribution parameters using bias and mean square error (MSE). First, we generate sample sizes from *X* ≈ Lindley (*θ*_1_) and *Y* ≈ Lindley (*θ*_2_) such as (*n*, *m*) = (5, 5), (10, 10), (30, 30), (50, 50), (100,100)  using different values of distribution parameters *X* and *Y* as (*θ*_1_, *θ*_2_) = (0.5,0.5), (0.5,1.5), (2,0.5), (1.5,1.5). For the Bayesian estimator, using noninformative prior and informative prior with parameters *a*_1_ = 3, *b*_1_ = 4, *a*_2_ = 2, *b*_2_ = 3, the results of this simulation study are shown in Tables 1–6

Table 1 shows that for both MLE and MPS for *R* and MRS, the MSE is decreasing when the sample size increases. In the context of comparison between estimates in almost all cases in Table 1, the MSE for MPS is smaller than MSE for MLE.  Table 2 shows that in the Bayesian estimates using MCMC and IS for *R* and MRS, the MSE is decreasing when the sample size increases. In the context of comparison between estimates in almost all cases in Table 2, the MSE for IS smaller than MSE for MCMC. Also, in the context of comparison between Bayesian and non-Bayesian estimates for *R* and MRS, in almost all cases, we get that the MSE in Bayesian estimates is smaller than MSE in non-Bayesian estimates. Tables 3–6 show the Bayesian and non-Bayesian estimators of FSS and FMRS for different values of parameters, sample sizes, and *k*.  Table 3 shows the results of MLE and MPS for FSS and FMRS when *θ*_1_ = *θ*_2_ = 0.5 and *k* = 1, 5, 10, 20. In general, the MSE decreases when the sample size increases. Also, the MSE for MPS estimator is smaller than the MSE for MLE. The MSE when *k* = 1 is smaller than MSE for another value of *k*. In Table 1 and Table 3, we get that the MSEs for *R* and MRS are smaller than the MSEs for FSS and FMRS.  Table 4 shows the results of Bayesian estimators for FSS and FMRS; in general, the MSE decreases when the sample size increases, but the MSE for IS method is smaller than the MSE for MCMC method; but the MSE for large *k* is smaller than the MSE for small *k*. In Table 2 and Table 4, we get that the MSEs for *R* and MRS are smaller than the MSEs for FSS and FMRS.  Table 5 and Table 6 show the non-Bayesian and Bayesian estimators for FSS and FMRS for other values of distribution parameters.

The article "Fuzzy Stress-Strength Model and Mean Remaining Strength for Lindley Distribution: Estimation and Application in Cancer of Benign Endocrine" was published in 2023. Journal: Comput Math Methods Med.

## 6. Medical Application (Cancer of Benign Endocrine)

The National Cancer Registration and Analysis Service (NCRAS) presents the numbers and percentages of tumors diagnosed in England in 2013-2018 recorded as receiving radiotherapy, chemotherapy, or tumor resection. In this study, we are more interested in the effectiveness of radiotherapy in diagnosing the benign endocrine cancer than chemotherapy. To investigate this aim, we use the data from NCRAS, as follows: the first data set *X* is the number of benign endocrine tumors which are diagnosed by radiotherapy, and the second data set *Y* is the number of benign endocrine tumors which are diagnosed by chemotherapy. The first and second data sets are defined in Table 7.

First, we must prove that the Lindley distribution is a good fit for two data sets; for this aim, we use the Anderson-Daring test, Cramer-Von Mises test, and *Q*-*Q* plot.  Table 8 and Figure 6 show that the Lindley distribution is a good fit for two data sets. In Table 8, we get the *p* value for two goodness of fit tests for two data sets more than 0.05, so the Lindley distribution is a good fit for two data sets.

In Table 9, we get that the classical estimators are greater than the fuzzy estimators. Also, for a large value of *k*, the fuzzy estimators are approximately equal to the classical estimators.

## 7. Conclusion

This study considers the stress-strength model and mean remaining strength using classical and fuzzy approaches when the stress and strength random variables are independent and have the Lindley distribution with different shape parameters. For non-Bayesian estimators, two estimation methods are used maximum likelihood and maximum product of spacing method. For Bayesian estimators, two algorithms are used Monte Carlo Markov Chain algorithm and the importance sampling algorithm. To compare between different estimators, simulation studies are performed. In general, the mean square error is decreasing when the sample size is increasing. To show the validity of our proposed models in real life, we apply our proposed model in the medical field. In the future, we want to use more recent data, get interval estimation, and also use more reliable models.

The article "Fuzzy Stress-Strength Model and Mean Remaining Strength for Lindley Distribution: Estimation and Application in Cancer of Benign Endocrine" was published in 2023. Journal: Comput Math Methods Med.

## Figures and Tables

**Figure 1:** Probability density function of the Lindley distribution when 0 < *θ* < 1.

**Figure 2:** Probability density function of the Lindley distribution when *θ* ≥ 1.

**Figure 3:** The mean residual function of the Lindley distribution.

**Figure 4:** The classical stress-strength model based on the Lindley distribution and different values of *θ*_1_ and *θ*_2_.

**Figure 5:** The fuzzy stress-strength model based on the Lindley distribution and different values of *k*, *θ*_1_ and *θ*_2_.

**Figure 6:** *Q*-*Q* plot for two data sets.

**Table 1:** Bias and MSE for maximum likelihood estimates and maximum product of spacing estimates of reliability parameter.

Sample size	MLE						MPS					
	$\hat{R}$	Bias	MSE	$\hat{\text{MRE}}$	Bias	MSE	*R* ^MPS^	Bias	MSE	MRE^MPS^	Bias	MSE
*θ*_1_ = 0.5, *θ*_2_ = 0.5, R_true_ = 0.5, MRS_True_ = 2.8889												
(5)	0.4406	-0.0059	0.0003	1.4230	-0.1465	0.2147	0.5591	0.0059	0.0003	3.7414	0.0852	0.0727
(10)	0.9201	0.0210	0.0088	2.3974	-0.0245	0.0121	0.4898	-0.0005	5.1 × 10^−6^	2.4788	-0.0204	0.0084
(30, 30)	0.9460	0.0071	0.0030	0.7930	-0.0349	0.0732	0.4726	-0.0004	0.1 × 10^−3^	2.7755	-0.0018	0.0002
(50, 50)	0.5259	0.0002	6.7 × 10^−6^	2.7242	-0.0016	0.0003	0.5744	0.0007	0.5 × 10^−4^	3.4208	0.0053	0.0028
(100, 100)	0.4542	-0.0002	0.1 × 10^−6^	2.3597	-0.0002	0.0001	0.4895	-0.5 × 10^−4^	5.4 × 10^−7^	2.9282	0.0001	7.7 × 10^−6^

*θ*_1_ = 0.5, *θ*_2_ = 1.5, R_true_ = 0.825, MRS_True_ = 3.0909												
(5)	0.7143	-0.0110	0.0012	1.4744	-0.1616	0.2612	0.9688	0.00143	0.0020	5.1230	0.2033	0.4733
(10)	0.7308	-0.0047	0.0044	2.2582	-0.0402	0.0324	0.8123	-0.0006	7.9 × 10^−6^	3.9000	0.0404	0.0327
(30, 30)	0.4872	-0.0056	0.0019	0.7609	-0.0388	0.0904	0.7420	-0.0013	0.0001	2.6626	-0.0071	0.0030
(50, 50)	0.8556	0.0006	0.1 × 10^−3^	2.9229	-0.0016	0.0002	0.7882	-0.0003	1 × 10^−4^	3.0208	0.0007	0.4 × 10^−4^
(100, 100)	0.7871	-0.0001	7.1 × 10^−6^	2.5054	-0.0029	0.0017	0.8503	0.0001	3.2 × 10^−6^	3.6667	0.0028	0.1 × 10^−6^

*θ*_1_ = 2, *θ*_2_ = 0.5, R_true_ = 0.1253, MRS_True_ = 0.6241												
(5)	0.2895	0.0164	0.0027	0.8192	0.0195	0.0038	0.1455	0.0020	0.4 × 10^−4^	0.9277	0.0303	0.0092
(10)	0.7701	0.0322	0.0207	0.8790	0.0127	0.0034	0.1150	-0.0005	5.2 × 10^−6^	0.4629	-0.0081	0.0012
(30, 30)	0.9114	0.0131	0.0103	0.6784	.0009	0.4 × 10^−4^	0.0977	-0.0004	0.1 × 10^−4^	0.6643	0.0007	0.2 × 10^−4^
(50, 50)	0.1645	0.0003	1 × 10^−5^	0.6877	0.0006	0.4 × 10^−4^	0.1604	0.0003	0.1 × 10^−4^	0.7097	0.0008	0.7 × 10^−4^
(100, 100)	0.1362	0.0001	5.9 × 10^−7^	0.6287	0.2 × 10^−4^	1.09 × 10^−7^	0.1385	0.6 × 10^−4^	8.7 × 10^−7^	0.7260	0.0005	0.5 × 10^−4^

*θ*_1_ = 1.5, *θ*_2_ = 1.5, R_true_ = 0.5, MRS_True_ = 2.8889												
(5)	0.6397	0.0139	0.0019	1.0792	-0.1780	0.3171	0.5648	0.0064	0.0004	0.8432	-0.2045	0.4184
(10)	0.5711	0.0036	0.0003	1.2828	-0.0802	0.1289	0.6128	0.0056	0.0006	1.0218	-0.0933	0.1742
(30, 30)	0.5526	0.0008	4 × 10^−5^	0.9547	-0.0322	0.0623	0.0977	-0.0067	0.0026	0.6643	-0.0371	0.0824
(50, 50)	0.6207	0.0012	0.0001	1.0397	-0.0184	0.0341	0.5813	0.0008	0.6×10^−4^	0.9131	-0.0197	0.0390
(100, 100)	0.5308	0.0001	4.7 × 10^−6^	0.9516	-0.0096	0.0187	0.5093	0.4 × 10^−4^	4.3 × 10^−7^	0.8747	-0.0100	0.0202

The article "Fuzzy Stress-Strength Model and Mean Remaining Strength for Lindley Distribution: Estimation and Application in Cancer of Benign Endocrine" was published in 2023. Journal: Comput Math Methods Med.

**Table 2:** Bias and MSE for Bayesian estimates of reliability parameter *R* = *P*[*Y* < *X*] and mean remaining strength.

Sample size	MCMC						IS					
	$\hat{R}$	Bias	MSE	$\hat{\text{MRE}}$	Bias	MSE	R^MPS^	Bias	MSE	MRE^MPS^	Bias	MSE
*θ*_1_ = 0.5, *θ*_2_ = 0.5, R_true_ = 0.5, MRS_True_ = 2.8889, a_1_ = 3, b_1_ = 4, a_2_ = 2, b_2_ = 3												
(5)	0.4989	-0.0001	1.1 × 10^−7^	1.3736	-0.1515	0.2295	0.5012	0.0001	1.48 × 10^−7^	1.3961	-0.1492	0.2227
(10)	0.4993	−0.3 × 10^−4^	1.9 × 10^−8^	1.3768	-0.0755	0.1142	0.5008	4 × 10^−4^	4 × 10^−8^	1.3846	-0.0752	0.1131
(30, 30)	0.5002	3.4 × 10^−6^	7.8 × 10^−10^	1.3751	-0.02252	0.0381	0.4985	−0.2 × 10^−4^	3.3 × 10^−8^	1.3761	-0.0252	0.0381
(50, 50)	0.4983	−0.1 × 10^−4^	2.7 × 10^−8^	1.3732	-0.0151	0.0229	0.4986	−0.1 × 10^−4^	1.8 × 10^−8^	1.3737	-0.0151	0.0229
(100, 100)	.4986	−6.8 × 10^−4^	9.4 × 10^−9^	1.3722	-0.0075	0.0114	0.4983	−8.4 × 10^−8^	1.4 × 10^−8^	1.3717	-0.0075	0.0115

*θ*_1_ = 0.5, *θ*_2_ = 1.5, R_true_ = 0.825, MRS_True_ = 3.0909a_1_ = 3, b_1_ = 4, a_2_ = 2, b_2_ = 3												
(5)	0.4987	-0.0326	0.0106	1.37414	-0.1719	0.2956	0.5067	-0.0318	0.0101	1.400	-0.1690	0.2859
(10)	0.5012	-0.0160	0.0052	1.3736	-0.0858	0.0474	0.5013	-0.0161	0.0052	1.3844	-0.0853	0.1456
(30, 30)	0.4991	-0.0054	0.0017	1.3720	-0.0286	0.0049	0.5012	-0.0053	0.0017	1.3810	-0.0284	0.0487
(50, 50)	0.5002	-0.0032	0.0010	1.3762	-0.0171	0.0294	0.5007	-0.0032	0.0010	1.3804	-0.0171	0.0292
(100, 100)	0.5003	-0.0016	0.0005	1.3776	-0.0085	0.0146	0.5006	-0.0016	0.0005	1.3767	-0.0085	0.0146

*θ*_1_ = 2, *θ*_2_ = 0.5, R_true_ = 0.1253, MRS_True_ = 0.6241a_1_ = 3, b_1_ = 4, a_2_ = 2, b_2_ = 3												
(5)	0.5004	0.0375	0.0140	1.3755	0.0751	0.0564	0.4978	0.0372	0.0139	1.3797	0.0755	0.0571
(10)	0.4992	0.0186	0.0069	1.3695	0.0372	0.0277	0.4989	0.0186	0.0069	1.3805	0.0378	0.0286
(30, 30)	0.5000	0.0062	0.0023	1.3768	0.0125	0.0094	0.5001	0.0062	0.0023	1.3815	0.0126	0.0095
(50, 50)	0.5003	0.0037	0.0014	1.37792	0.0075	0.0057	0.4991	0.0037	0.0013	1.3744	0.0075	0.0056
(100, 100)	0.4996	0.0018	0.0007	1.3737	0.0037	0.0028	0.5011	0.0018	0.0007	1.3800	0.0037	0.0028

*θ*_1_ = 1.5, *θ*_2_ = 1.5, R_true_ = 0.5, MRS_True_ = 2.8889a_1_ = 3, b_1_ = 4, a_2_ = 2, b_2_ = 3												
(5)	0.5012	0.0001	1.6 × 10^−7^	1.3795	-0.1509	0.2277	0.4986	-0.0001	1.7 × 10^−7^	1.3796	-0.1508	0.2275
(10)	0.5008	0.4 × 10^−4^	3.3 × 10^−8^	1.3757	-0.0756	0.1144	0.4996	−0.1 × 10^−4^	4.8 × 10^−9^	1.3806	-0.0755	0.1136
(30, 30)	0.5000	1.14 × 10^−6^	7.9 × 10^−8^	1.3784	-0.0251	0.0380	0.4997	−3.4 × 10^−6^	7.1 × 10^−10^	1.3777	-0.0251	0.0380
(50, 50)	0.4996	−3.7 × 10^−6^	1.4 × 10^−8^	1.3783	-0.0151	0.0229	0.4984	0.4 × 10^−4^	2.9 × 10^−10^	1.3752	-0.0151	0.0028
(100, 100)	0.4982	−8.6 × 10^−6^	1.4 × 10^−9^	1.3730	-0.0075	0.0114	0.4997	−1.2 × 10^−6^	2.5 × 10^−10^	1.3779	-0.0075	0.0114

The article "Fuzzy Stress-Strength Model and Mean Remaining Strength for Lindley Distribution: Estimation and Application in Cancer of Benign Endocrine" was published in 2023. Journal: Comput Math Methods Med.

**Table 3:** Bias and MSE for MLE and MPS estimate of reliability parameter FSS and FMRS.

Sample size	MLE						MPS					
	$\hat{\text{FSS}}$	Bias	MSE	$\text{F}\hat{\text{MRE}}$	Bias	MSE	FSS^MPS^	Bias	MSE	FMRE^MPS^	Bias	MSE
*θ*_1_ = 0.5, *θ*_2_ = 0.5, FSS_true_ = 0.3827, FMRS_True_ = 3.5268, *k* = 1												
(5)	0.2652	-0.0234	0.0055	1.9521	-0.0935	0.0875	0.4549	0.0072	0.0005	4.4004	0.0873	0.0763
(10)	0.2328	-0.0133	0.0035	2.7540	-0.0066	0.0008	0.3595	-0.0011	0.2 × 10^−4^	3.0975	-0.0214	0.0092
(30, 30)	0.4177	-0.0013	0.0001	1.1918	-0.0282	0.0479	0.3577	-0.0004	0.1 × 10^−4^	3.4110	-0.0019	0.0002
(50, 50)	0.3967	-0.0010	0.0001	3.3524	0.0046	0.0021	0.4587	0.0007	0.5 × 10^−4^	4.0694	0.0054	0.0029
(100, 100)	0.3283	-0.0008	0.0001	2.9741	0.0004	3 × 10^−4^	0.3759	−0.3 × 10^−4^	2.2 × 10^−4^	3.5688	0.0002	8.8 × 10^−6^

*θ*_1_ = 0.5, *θ*_2_ = 0.5, FSS_true_ = 0.4729, FMRS_True_ = 3.0432, *k* = 5												
(5)	0.3915	-0.0108	0.0011	1.5789	-0.1309	0.1713	0.5363	0.0063	0.0004	3.8924	0.0849	0.0721
(10)	0.3076	-0.0096	0.0018	2.3052	-0.0291	0.0169	0.4587	-0.0007	0.1 × 10^−4^	2.6339	-0.0204	0.0083
(30, 30)	0.7513	0.0041	0.0010	0.9372	-0.0325	0.0634	0.4457	-0.0004	10.1 × 0^−4^	2.9308	-0.0018	0.0002
(50, 50)	0.4958	−0.4 × 10^−4^	1.7 × 10^−7^	2.8779	-0.0001	1 × 10^−6^	0.5487	0.0007	0.5 × 10^−4^	3.5717	0.0052	0.0027
(100, 100)	0.4237	-0.0003	0.2 × 10^−4^	2.5158	-0.0018	0.0006	0.4633	−0.4 × 10^−4^	4.5 × 10^−7^	3.0828	0.0001	7.8 × 10^−6^

*θ*_1_ = 0.5, *θ*_2_ = 0.5, FSS_true_ = 0.4862, FMRS_True_ = 2.9676, *k* = 10												
(5)	0.4149	-0.0085	0.0007	1.5054	-0.1382	0.1911	0.5476	0.0061	0.0003	3.8179	0.085	0.0723
(10)	0.3198	-0.0090	0.0016	2.2285	-0.0329	0.0217	0.474	-0.0006	7.4 × 10^−6^	2.5583	-0.0204	0.0083
(30, 30)	0.8305	0.0055	0.0018	0.8724	-0.0335	0.0677	0.4589	-0.0004	0.1 × 10^−4^	2.8549	-0.0018	0.0002
(50, 50)	0.5106	0.0001	1.13 × 10^−6^	2.8027	-0.0008	0.7 × 10^−4^	0.5615	0.0007	0.5 × 10^−4^	3.4973	0.0052	0.0028
(100, 100)	0.4386	-0.0003	0.1 × 10^−4^	2.4400	-0.0022	0.0010	0.4762	−0.4 × 10^−4^	4.9 × 10^−7^	3.0071	0.0001	7.8 × 10^−6^

*θ*_1_ = 0.5, *θ*_2_ = 0.5, FSS_true_ = 0.4930, FMRS_True_ = 2.9286, *k* = 20												
(5)	0.4274	-0.0072	0.0005	1.4655	-0.1422	0.2023	0.5533	0.006	0.0003	3.7799	0.0851	0.0724
(10)	0.3261	-0.0086	0.0015	2.1881	-0.0344	0.0244	0.4818	-0.0005	6.1 × 10^−6^	2.519	-0.0204	0.0083
(30, 30)	0.8756	0.0062	0.0023	0.8347	-0.0342	0.0702	0.4657	-0.0004	0.1 × 10^−4^	2.8156	-0.0018	0.0002
(50, 50)	0.5182	0.0001	3.3 × 10^−6^	2.7639	-0.0012	0.0015	0.5679	0.0007	0.5 × 10^−4^	3.4593	0.0053	0.0028
(100, 100)	0.4463	-0.0002	0.1 × 10^−4^	2.4004	-0.0024	0.0011	0.4828	−0.5 × 10^−4^	5.1 × 10^−7^	2.968	0.0001	7.8 × 10^−6^

The article "Fuzzy Stress-Strength Model and Mean Remaining Strength for Lindley Distribution: Estimation and Application in Cancer of Benign Endocrine" was published in 2023. Journal: Comput Math Methods Med.

**Table 4:** Bias Bayesian estimate of reliability parameter FSS and FMRS.

Sample size	MCMC						IS					
	$\hat{\text{FSS}}$	Bias	MSE	$\text{F}\hat{\text{MRE}}$	Bias	MSE	FSS^MPS^	Bias	MSE	FMRE^MPS^	Bias	MSE
*θ*_1_ = 0.5, *θ*_2_ = 0.5, FSS_true_ = 0.3827, FMRS_True_ = 3.5268, *k* = 1												
(5)	0.2961	-0.0086	0.0007	1.8932	-0.1674	0.2804	0.2995	-0.0083	0.0006	1.9187	-0.1649	0.2719
(10)	0.2966	-0.0043	0.0003	1.8968	-0.0835	0.1396	0.2983	-0.0042	0.0003	1.9056	-0.0831	0.1381
(30, 30)	0.2970	-0.0014	0.0001	1.8949	-0.0278	0.0466	0.2961	-0.00086	0.7 × 10^−4^	1.8960	-0.0167	0.0279
(50, 50)	0.2957	-0.0008	0.7 × 10^−4^	1.8927	-0.0167	0.0280	0.2965	-0.0008	0.7 × 10^−4^	1.8934	-0.0167	0.0280
(100, 100)	0.2957	-0.0004	0.3 × 10^−4^	1.8916	-0.0083	0.0140	0.2955	-0.0004	0.3 × 10^−4^	1.891	-0.0083	0.0140

*θ*_1_ = 0.5, *θ*_2_ = 0.5, FSS_true_ = 0.4729, FMRS_True_ = 3.0432, *k* = 5												
(5)	0.4417	-0.0031	0.9 × 10^−4^	1.5280	-0.1515	0.2295	0.4446	-0.0028	0.7 × 10 − 4	1.5506	-0.1492	0.2227
(10)	0.4422	0.0015	0.4 × 10^−4^	1.5312	-0.0755	0.11429	0.4438	-0.0014	0.4 × 10^−4^	1.539	-0.0752	0.1131
(30, 30)	0.4428	-0.0005	0.1 × 10^−4^	1.5295	-0.0252	0.0381	0.4414	-0.0005	0.1 × 10^−4^	1.5305	-0.0252	0.0381
(50, 50)	0.4411	-0.0003	0.1 × 10^−4^	1.5276	-0.0151	0.0229	0.4414	-0.0003	9.8 × 10^−6^	1.5281	0.0151	0.0229
(100, 100)	0.4413	-0.0001	4.9 × 10^−6^	1.5266	-0.0075	0.01149	0.4410	-0.0001	5 × 10^−6^	1.5261	-0.0075	0.0115

*θ*_1_ = 0.5, *θ*_2_ = 0.5, FSS_true_ = 0.4862, FMRS_True_ = 2.9676, *k* = 10												
(5)	0.4690	-0.0017	0.2 × 10^−4^	1.4551	-0.1512	0.2287	0.4716	-0.0014	0.2 × 10^−4^	1.4776	-0.1489	0.2219
(10)	0.4694	-0.0008	0.1 × 10^−4^	1.4583	-0.0754	0.1138	0.4711	-0.0007	0.1 × 10^−4^	1.4661	-0.0750	0.1127
(30, 30)	0.4702	-0.0002	4.2 × 10^−6^	1.4567	-0.0251	0.0380	0.4687	-0.0002	5 × 10^−6^	1.4576	-0.0251	0.0379
(50,50)	0.4684	-0.0001	3.1 × 10^−6^	1.4548	-0.0151	0.0228	0.4687	-0.0001	3 × 10^−6^	1.4553	-0.0151	0.0228
(100, 100)	0.4686	-0.0001	3 × 10^−6^	1.4538	-0.0151	0.0229	0.4683	-0.0001	3 × 10^−6^	1.4533	-0.0151	0.0229

*θ*_1_ = 0.5, *θ*_2_ = 0.5, FSS_true_ = 0.4930, FMRS_True_ = 2.9286, *k* = 20												
(5)	0.4833	-0.0009	9.2 × 10^−6^	1.4154	-0.1513	0.2289	0.4861	-0.0006	4.7 × 10^−6^	1.4380	-0.1490	0.2221
(10)	0.4841	-0.0004	3.9 × 10^−6^	1.4187	-0.0754	0.1139	0.4856	-0.0003	2.7 × 10^−6^	1.4265	-0.0751	0.1128
(30, 30)	0.4848	-0.0001	1 × 10^−6^	1.4170	-0.0251	0.0380	0.4833	-0.0001	1.5 × 10^−6^	1.4180	-0.0251	0.0380
(50, 50)	0.4830	−0.9 × 10^−4^	9.8 × 10^−7^	1.4151	-0.0151	0.0229	0.4833	−0.9 × 10^−4^	9.8 × 10 − 7	1.4156	-0.0151	0.0228
(100, 100)	0.4833	−0.4 × 10^−4^	4.7 × 10^−7^	1.4141	-0.0075	0.0114	0.4830	−0.4 × 10^−4^	4.9 × 10^−7^	1.4136	-0.0075	0.0114

The article "Fuzzy Stress-Strength Model and Mean Remaining Strength for Lindley Distribution: Estimation and Application in Cancer of Benign Endocrine" was published in 2023. Journal: Comput Math Methods Med.

**Table 5:** Bias and MSE for MLE and MPS estimate of reliability parameter FSS and FMRS.

Sample size	MLE						MPS					
	$\hat{\text{FSS}}$	Bias	MSE	$\text{F}\hat{\text{MRE}}$	Bias	MSE	FSS^MPS^	Bias	MSE	FMRE^MPS^	Bias	MSE
*θ*_1_ = 0.5, *θ*_2_ = 1.5, FSS_true_0.65, FMRS_True_ = 3.6923, *k* = 1												
(5)	0.4388	-0.0211	0.00445	1.9966	-0.1695	0.2875	0.8546	0.0204	0.0041	5.6835	0.1991	0.3965
(100, 100)	0.5850	-0.0003	0.2 × 10^−4^	3.0944	-0.0029	0.0017	0.6976	0.0002	0.1 × 10^−4^	4.2718	0.0028	0.0016

*θ*_1_ = 0.5, *θ*_2_ = 1.5, FSS_true_ = 0.7871, FMRS_True_ = 3.2297, *k* = 5												
(5)	0.6396	-0.0147	0.0021	1.6252	-0.1604	0.2574	0.9482	0.0161	0.0025	5.2417	0.2012	0.4048
(100, 100)	0.7408	-0.0046	0.0002	2.6492	-0.0580	0.0336	0.8187	0.0031	0.0001	3.8006	0.0570	0.0325

*θ*_1_ = 0.5, *θ*_2_ = 1.5, FSS_true_ = 0.8061, FMRS_True_ = 3.1609, *k* = 10												
(5)	0.6756	-0.0130	0.0017	1.5534	-0.1607	0.2583	0.9587	0.0152	0.0023	5.1765	0.2015	0.4062
(100, 100)	0.7618	-0.0002	9.8 × 10^−6^	2.5572	-0.0030	0.0018	0.8346	0.0001	4.1 × 10^−6^	3.7338	0.0028	0.0016

*θ*_1_ = 0.5, *θ*_2_ = 1.5, FSS_true_ = 0.8155, FMRS_True_ = 3.1260, *k* = 20												
(5)	0.4655	−0.0349	0.0122	1.4717	−0.1684	0.2836	0.9639	0.01484	0.0022	5.1603	0.2004	0.4017
(100, 100)	0.7754	−0.0002	8 × 10^−6^	2.5419	−0.0030	0.0018	0.8425	0.0001	3.6 × 10^−6^	3.7002	0.0027	0.0014

*θ*_1_ = 2, *θ*_2_ = 0.5, FSS_true_ = 0.0486, FMRS_True_ = 0.9871, *k* = 1												
(5)	0.1314	0.0082	0.0006	1.2381	0.0251	0.0063	0.0711	0.0022	0.5 × 10^−4^	1.3763	0.0389	0.0151
(100, 100)	0.0531	0.2 × 10^−4^	1.1 × 10^−7^	0.9932	0.3 × 10^−4^	1.9 × 10^−7^	0.0590	0.5 × 10^−4^	5.4 × 10^−7^	1.1212	0.0006	0.9 × 10^−4^

*θ*_1_ = 2, *θ*_2_ = 0.5, FSS_true_ = 0.0958, FMRS_True_ = 0.7682, *k* = 5												
(5)	0.2337	0.0137	0.0019	0.9691	0.0201	0.0040	0.1210	0.0025	0.6 × 10^−4^	1.0811	0.0312	0.0097
(100, 100)	0.1044	0.4 × 10^−4^	3.7 × 10^−7^	0.7730	0.2 × 10^−4^	1.2 × 10^−7^	0.1097	0.6 × 10^−4^	9.8 × 10^−7^	0.8741	0.0005	0.5 × 10^−4^

*θ*_1_ = 2, *θ*_2_ = 0.5, FSS_true_ = 0.1087, FMRS_True_ = 0.7058, *k* = 10												
(5)	0.2581	0.0149	0.0022	0.9018	0.0196	0.0038	0.0038	0.0023	0.5 × 10^−4^	1.0114	0.0305	0.0093
(100, 100)	0.1183	0.4 × 10^−4^	4.6 × 10^−7^	0.7105	0.2 × 10^−4^	1.1 × 10^−7^	0.1226	0.6 × 10^−4^	9.7 × 10^−7^	0.8086	0.0005	0.5 × 10^−4^

*θ*_1_ = 2, *θ*_2_ = 0.5, FSS_true_ = 0.1165, FMRS_True_ = 0.6678, k =20												
(5)	0.2721	0.0155	0.00242	0.8626	0.0194	0.0037	0.1386	0.0022	0.4 × 10^−4^	0.9715	0.0303	0.0092
(100, 100)	0.1397	0.0001	2.7 × 10^−6^	0.6731	0.2 × 10^−4^	1.4 × 10^−7^	0.1301	0.6 × 10^−4^	9.3 × 10^−7^	0.7697	0.0005	0.5 × 10^−4^

The article "Fuzzy Stress-Strength Model and Mean Remaining Strength for Lindley Distribution: Estimation and Application in Cancer of Benign Endocrine" was published in 2023. Journal: Comput Math Methods Med.

**Table 6:** Bias Bayesian estimate of reliability parameter FSS and FMRS.

Sample size	MCMC						IS					
	$\hat{\text{FSS}}$	Bias	MSE	$\text{F}\hat{\text{MRE}}$	Bias	MSE	FSS^MPS^	Bias	MSE	FMRE^MPS^	Bias	MSE
*θ*_1_ = 0.5, *θ*_2_ = 1.5, FSS_true_0.65, FMRS_True_ = 3.6923, *k* = 1												
(5)	0.2956	-0.0354	0.0125	1.8907	-0.1801	0.3245	0.3032	-0.0346	0.0120	1.9229	-0.1769	0.3130
(100, 100)	0.2973	-0.0017	0.0006	1.8976	-0.0089	0.0161	0.2974	-0.0017	0.0006	1.8967	-0.0089	0.0161

*θ*_1_ = 0.5, *θ*_2_ = 1.5, FSS_true_ = 0.7871, FMRS_True_ = 3.2297, *k* = 5												
(5)	0.4412	0.0345	0.0119	1.5258	-0.1703	0.2902	0.4496	-0.0337	0.0113	1.5544	-0.1675	0.2806
(100, 100)	0.4430	-0.0344	0.0118	1.5320	-0.1697	0.2882	0.4433	-0.0343	0.0118	1.5311	-0.1698	0.2885

*θ*_1_ = 0.5, *θ*_2_ = 1.5, FSS_true_ = 0.8061, FMRS_True_ = 3.1609, *k* = 10												
(5)	0.4685	-0.0337	0.0113	1.4530	-0.1707	0.2916	0.4769	-0.0329	0.0108	1.4814	-0.1679	0.2820
(100, 100)	0.4703	-0.0016	0.0005	1.4591	-0.0085	0.0144	0.4706	-0.0016	0.0005	1.4582	0.0085	0.0144

*θ*_1_ = 0.5, *θ*_2_ = 1.5, FSS_true_ = 0.8155, FMRS_True_ = 3.1260, *k* = 20												
(5)	0.4831	-0.0332	0.0110	1.4133	-0.1742	0.3036	0.4915	-0.0323	0.0104	1.4418	-0.1714	0.2938
(100, 100)	0.4850	-0.0016	0.0005	1.4194	-0.0086	0.0150	0.4853	-0.0016	0.0005	1.4186	-0.0086	0.0151

*θ*_1_ = 2, *θ*_2_ = 0.5, FSS_true_ = 0.0486, FMRS_True_ = 0.9871, *k* = 1												
(5)	0.2972	0.0248	0.0061	1.8953	0.0908	0.0824	0.2960	0.0247	0.0061	1.9002	0.0913	0.0833
(100, 100)	0.2965	0.0012	0.0003	1.8933	0.0045	0.0041	0.2980	0.0012	0.0003	1.9003	0.0045	0.0041

*θ*_1_ = 2, *θ*_2_ = 0.5, FSS_true_ = 0.0958, FMRS_True_ = 0.7682, *k* = 5												
(5)	0.4431	0.0347	0.0121	1.5299	0.0761	0.0580	0.4409	0.0345	0.0119	1.5342	0.0766	0.0586
(100, 100)	0.4423	0.0017	0.0006	1.5281	0.0037	0.0028	0.4439	0.0017	0.0006	1.5344	0.0038	0.0029

*θ*_1_ = 2, *θ*_2_ = 0.5, FSS_true_ = 0.1087, FMRS_True_ = 0.7058, *k* = 10												
(5)	0.4705	0.0361	0.0131	1.4571	0.0751	0.0564	0.4681	0.0359	0.0129	1.4613	0.0755	0.0571
(100, 100)	0.4697	0.0018	0.0006	1.4553	0.0037	0.0028	0.4712	0.0018	0.0006	1.4615	0.0037	0.0028

*θ*_1_ = 2, *θ*_2_ = 0.5, FSS_true_ = 0.1165, FMRS_True_ = 0.6678, *k* = 20												
(5)	0.4851	0.0368	0.0135	1.4174	0.0749	0.0561	0.4826	0.0366	0.0134	1.4216	0.0753	0.0568
(100, 100)	0.4843	0.0018	0.0006	1.4156	0.0037	0.0027	0.4858	0.0018	0.0006	1.4218	0.0037	0.0028

The article "Fuzzy Stress-Strength Model and Mean Remaining Strength for Lindley Distribution: Estimation and Application in Cancer of Benign Endocrine" was published in 2023. Journal: Comput Math Methods Med.

**Table 7:** Cancer of benign endocrine dataset.

Data set I (*X*)	6	6	7	3	3	4	1	50	7	9	13	14	16	31	28	59	13	13	11	9	12	9	5	
Data set II (*Y*)	1	1	1	3	3	1	1	18	4	5	6	6	4	5	5	9	15	24	4	2	5	5	7	1

**Table 8:** The result of goodness of fit tests.

Data set	Test	Statistic	*p* value
Data set I	Anderson-Daring	1.0397	0.1050
	Cramer-Von Mises	0.1834	0.0874

Data set II	Anderson-Daring	1.1327	0.0814
	Cramer-Von Mises	0.1556	0.1332

**Table 9:** The results of our proposed estimators for two data sets.

Estimation method	*R*	MRS	FSS				FMRS			
			*k* = 1	*k* = 5	*k* = 10	*k* = 20	*k* = 1	*k* = 5	*k* = 10	*k* = 20
MLE	0.8544	5.3576	0.7999	0.8339	0.8444	0.8494	5.9686	5.4840	5.4205	5.3889
MPS	0.7848	12.9964	0.7454	0.7772	0.7811	0.7830	13.6294	13.1221	13.0591	13.0276
MCMC	0.4994	1.3758	0.2966	0.4422	0.4695	0.4841	1.8956	1.5302	1.4573	1.4176
IS	0.5015	1.3784	0.2981	0.4422	0.4715	0.4862	1.8985	1.5328	1.4599	1.4202

## Data Availability

The data used to support the findings of this study are included within the article.

## Abbreviations

IS: Importance sampling
MH: Metropolis-Hastings
MPS: Maximum product of spacing
MLE: Maximum likelihood estimation
MRS: Mean remaining strength
MCMC: Monte Carlo Markov chain
FSS: Fuzzy stress-strength model
FMRS: Fuzzy mean remaining strength
MSE: Mean square error.
